The article "Combined Network Pharmacology and Molecular Docking to Verify the Treatment of Type 2 Diabetes with Pueraria Lobata Radix and Salviae Miltiorrhizae Radix" was published in 2023. Journal: Comput Math Methods Med.

# Combined Network Pharmacology and Molecular Docking to Verify the Treatment of Type 2 Diabetes with *Pueraria Lobata Radix* and *Salviae Miltiorrhizae Radix*

**DOI:** 10.1155/2023/9150324

**Published:** 2023-02-11

**Authors:** Jingxin Mao, Guowei Wang, Lin Yang, Lihong Tan, Cheng Tian, Lijing Tang, Ling Fang, Zhenqiang Mu, Zhaojing Zhu, Yan Li

**Affiliations:** ^1^Chongqing Medical and Pharmaceutical College, Chongqing 400030, China; ^2^College of Pharmaceutical Sciences, Southwest University, Chongqing 400715, China; ^3^Chongqing Key Laboratory of High Active Traditional Chinese Drug Delivery System, Chongqing 400030, China

## Abstract

**Objective:**

To explore the potential molecular mechanism of *Pueraria Lobata Radix* (RP) and *Salviae Miltiorrhizae Radix* (RS) in the treatment of type 2 diabetes mellitus (T2DM) based on network pharmacology and molecular docking.

**Methods:**

The chemical constituents and core targets of RP and RS were searched by Traditional Chinese Medicine System Pharmacology (TCMSP); target genes related to T2DM were obtained through GeneCards database, component target network diagram was constructed, intersection genes of active compounds and T2DM were synthesized, protein-protein interaction (PPI) relationship was obtained, and core targets were screened by using Cytoscape 3.7.2. Gene Ontology (GO) biological process and Kyoto Encyclopedia of Genes and Genomes (KEGG) pathway were analyzed utilizing R studio 4.0.4 according to David database. Based on molecular docking, the screened active components of RP and RS were verified by molecular docking with the core target using Discovery Studio 2019.

**Results:**

There were totally 92 components and 29 corresponding targets in the component target network of RP and RS drug pair, of which 6 were the core targets of RP and RS in the treatment of T2DM. Molecular docking results showed that the active compounds of puerarin, formononetin, tanshinone iia, and luteolin had better binding activity with AKT1, VEGFA, NOS3, PPARG, MMP9, and VCAM1, respectively. Among them, puerarin showed significant effects in activating NOS3 pathway and luteolin exhibited significant effects in activating MMP9 pathway, respectively. The main biological processes mainly including xenobiotic stimulus, response to peptide, gland development, response to radiation, cellular response to chemical stress, response to oxygen levels, and the main signal pathways include response to xenobiotic stimulus, cellular response to chemical stress, response to peptide, gland development, and response to oxygen levels.

**Conclusion:**

Network pharmacology is an effective tool to explain the action mechanism of Traditional Chinese Medicine (TCM) from the overall perspective. RP and RS pair could alleviate T2DM via the molecular mechanism predicted by the network pharmacology, which provided new ideas and further research on the molecular mechanism of T2DM.

The article "Combined Network Pharmacology and Molecular Docking to Verify the Treatment of Type 2 Diabetes with Pueraria Lobata Radix and Salviae Miltiorrhizae Radix" was published in 2023. Journal: Comput Math Methods Med.

## 1. Introduction

Diabetes mellitus (DM) is a group of metabolic diseases characterized by increased blood glucose due to genetic and environmental effects, resulting in defective insulin secretion and reduced sensitivity of target cells to insulin. Type 2 diabetes mellitus (T2DM) is a chronic metabolic disease, mainly associated with the accumulation of lipids in the insulin *β*-cells can lead to elevated blood glucose levels and abnormal glucose tolerance due to the dysfunction of the pancreatic *β*-cells, and the clinical symptoms are persistent hyperglycemia. In recent decades, the prevalence of T2DM has gradually increased worldwide. The prevalence of DM in the world has increased by 102.9% from 1990 to 2010 and is the country with the largest number of diabetic patients in the world [1]. T2DM is a common clinical endocrine and metabolic disease, and the prevalence of DM in Chinese population is about 11.6%, and the prevalence of pre-DM is 50.1% [2], which is a chronic metabolic disease that seriously affects human health.

The important cause of T2DM is the disorder of lipid metabolism, therefore, it is especially important to control blood sugar and regulate blood lipid in the process of T2DM treatment in time [3]. At present, the main methods of T2DM drug treatment are subcutaneous insulin injection and oral hypoglycemic drugs (such as double pulse, sulfonyl artery, and a glyoxylase inhibitors); but with the development of the diseas

e, single-target development of drugs is difficult to treat T2DM and prevent the occurrence of complications such as glucose disorders and gastrointestinal tract, thus reducing the quality of life of patients [4].

Traditional Chinese Medicine (TCM) treatment of T2DM is based on single-target superposition and, multicomponent and multitarget synergistic toxicity dispersion effect to achieve better efficacy and lower toxicity group, which is a complex theoretical system to achieve multidimensional regulation from a whole [5]. DM belongs to the category of “thirst disorders” in TCM, and the main treatment of DM in TCM is to clear heat and moisten dryness, and to nourish yin and produce fluid [6]. After the TCM, doctors have formulated prescriptions according to the above treatment rules, the overall regulating advantages of TCM, which can play a role in treating both the symptoms and the root cause, and TCM is milder and more durable than western medicine, with fewer side effects [7].

The article "Combined Network Pharmacology and Molecular Docking to Verify the Treatment of Type 2 Diabetes with Pueraria Lobata Radix and Salviae Miltiorrhizae Radix" was published in 2023. Journal: Comput Math Methods Med.

*Pueraria Lobata Radix* (RP) and *Salviae Miltiorrhizae Radix* (RS) are a common pair of medicine contained in the famous Chinese medicine book “Shi Jinmo on Medicine.” RP is the dried root of *Pueraria lobata* (Willd.) Ohwi, which has the functions of quenching thirst, raising yang, relieving diarrhea, relieving muscle and fever, and activating meridians [8]. RS is also called “DanShen” that derived from the dried root and rhizome of *Salvia miltiorrhiza* Bunge, which has the effects of activating blood circulation, cooling the blood and clearing the heart, and removing irritation and calming the mind [9]. The combination of RP and RS exhibits the effect of promoting “qi,” resolving blood stasis, promoting blood circulation, and relieving pain, and the two are used as a pair to treat diabetes [10, 11]. Modern medicinal chemistry and pharmacology research shows that the main chemical components of RP are isoflavones, triterpenoids, flavonoids, coumarins, etc., which have pharmacological effects such as hypoglycemic and hypolipidemic, anti-inflammatory and antioxidant, and hepatoprotective [12]. The main chemical components of RS mainly including tanshinones, tanshin acids, and volatile oils, which have antioxidant, anti-inflammatory, and antithrombotic pharmacological effects [13].

Previous studies have been demonstrated that *Pueraria Lobata Radix* and *Salviae Miltiorrhizae Radix* (RP-RS) paired exhibits varies effects on T2DM or diabetes related diseases [10, 14–17]. However, the research on effective compounds of RP-RS is not in-depth, and the analytical methods are not comprehensive in these studies. Therefore, based on the idea of multicomponent and multitarget research, the present study was conducted to predict the mechanism of action and targets of RP-RS drug for the treatment of T2DM through network pharmacology and molecular docking methods, to find the active chemical components, disease therapeutic targets and signaling pathways, and to provide a scientific basis for the experimental research and clinical application of RP-RS drug for the treatment of T2DM.

## 2. Materials and Methods

### 2.1. Screening of RP and RS for Active Components and Potential Targets

The chemical components of RP and RS were obtained with the help of the Traditional Chinese Medicine System Pharmacology Analysis Platform (TCMSP, http://temspw.com/temsp.php), according to the set the bioavailability (OB) > 20 and drug-like properties (DL) > 0.18, screening out eligible active ingredients and related targets.

### 2.2. T2DM-Related Target Prediction

Through the GeneCards (http://www.genecards.org/) database, with “Type 2 diabetes mellitus or T2DM” as the search term, the targets related to T2DM were obtained, and the correlation value (relevance score > 18) was used as the screening condition, and the screening results were used as candidate target genes of T2DM.

The article "Combined Network Pharmacology and Molecular Docking to Verify the Treatment of Type 2 Diabetes with Pueraria Lobata Radix and Salviae Miltiorrhizae Radix" was published in 2023. Journal: Comput Math Methods Med.

### 2.3. Construction of Protein Interaction Network (PPI)

The effect of drugs on disease treatment is ultimately manifested in protein interactions. The Venn diagram (https://bioinfogp.cnb.csic.es/tools/venny/index.html) was used to obtain the intersection genes of the active ingredient target and the T2DM target, and imported into STRING11.0 (http://www.string-db.org/) to obtain the protein interaction relationship. Using Cytoscape 3.7.2 draws the interaction network, analyzes the key targets by degree value, and constructs the interaction network of RP-RS in the treatment of T2DM.

### 2.4. Construction of Chemical Components-Target Network of TCM

The screened candidate compounds of RP-RS that predicted component target genes were imported into Cytoscape 3.7.2 software to construct a compound-target network, and the main active ingredients/components of RP and RS were analyzed, respectively, according to the degree value in the network.

### 2.5. Analysis of Biological Function and Pathway Enrichment of RP-RS Pair in the Treatment of T2DM

GO enrichment is a commonly used method for analysis of omic data, which is usually used to discover the enrichment degree of GO term in differential genes. Through GO enrichment analysis, the genes in the difference table can be classified according to their functions to achieve the purpose of annotation and classification of genes [18]. KEGG is a practical program database for understanding advanced functions and biological systems (such as cells, organisms, and ecosystems) from molecular level information, especially genome sequencing and other high-throughput experimental technologies generated from large molecular data sets. It can predict the role of PPI networks in various cell activities [19]. Based on the David database (https://david.ncifcrf.gov/), the targets of RP-RS for the treatment of T2DM were collected and imported into R studio 4.0.4 (The species was limited to “Human”). GO functional annotation and KEGG pathway enrichment analysis were performed on the intersection target genes of RP-RS and T2DM, respectively (*P* < 0.05). Potential targets were analyzed for biological process (BP), cellular component (CC), and molecular function (MF), and KEGG was used for pathway enrichment analysis of potential targets. To validate the anti-T2DM mechanism of RP-RS across the key targets and multiple pathways, the KEGG mapper functional analysis was used to mark the target genes on the pathway associated with T2DM.

The article "Combined Network Pharmacology and Molecular Docking to Verify the Treatment of Type 2 Diabetes with Pueraria Lobata Radix and Salviae Miltiorrhizae Radix" was published in 2023. Journal: Comput Math Methods Med.

### 2.6. Molecular Docking Prediction of Key Targets of Active Ingredient Intervention in the Treatment of T2DM by RP-RS

According to the analysis of network pharmacology results, molecular docking software was used to predict the key targets of RP-RS intervention on the main active components. The 3D structure of the compound was constructed using Chem 3D of ChemOffice software and saved in.mol2 format. Download the protein structure of the target from the PDB (https://www.rcsb.org/) database, use PyMOL 2.5 to perform protein and ligand separation, dehydrogenation, water addition, and other operations on the original PDB protein molecule, and use AutoDock 1.5.7 software. The above compound and protein formats were converted to pdbqt format using Discovery Studio 2019 software for molecular docking and mapping of compounds and core targets.

## 3. Results

### 3.1. Screening of Active Compounds from RP-RS

Taking OB and DL properties as screening criteria, qualified compounds were screened from TCMSP database. After setting the screening conditions, 7 and 85 chemical components of RP and RS were obtained, respectively (Table 1).

### 3.2. Intersection Genes of RP-RS with T2DM

By database analysis, 356, 159, and 99 targets were identified for T2DM, RP, and RS, respectively. The online Venn diagram analysis showed that there were 28 intersecting genes between the active ingredient target of RS and T2DM (Figure 1(a)), 10 intersecting genes between the active ingredient target of RP and T2DM (Figure 1(b)), and 8 intersecting genes among RP, RS, and T2DM (Figure 1(c)), which were the main potential targets of RP-RS for the treatment of T2DM.

### 3.3. Protein Interaction PPI Network Construction

In this study, we analyzed the interaction between the targets of RP and RS for the treatment of T2DM based on the STRING database, and constructed the target interaction network (Figures 2(a) and 2(b)) by importing compound-disease shared genes into STRING with the interaction confidence setting, medium confidence (0.4), and performed the network topology analysis. The top 6 nodes in the interaction network were AKT1 (26), VEGFA (25), NOS3 (24), PPARG (22), MMP9 (22), and VCAM1 (20), (Table 2, Figure 2(b)), which may play an important role in the treatment of T2DM with RS. These 6 key targets may play an important role in the treatment of T2DM with RP.

### 3.4. Compound-Target Interaction Network

The network diagram visually reflects the interaction between compounds and targets, the nodes represent compounds, and the edges represent the relationship between compounds and targets, which can reflect the synergistic superposition of multicomponent and multitarget in Chinese medicine. The top 4 compounds in terms of degree value were MOL000006-luteolin (degree value = 54), MOL012297-puerarin (degree value = 53), MOL07154-tanshinone iia (degree value = 40), and MOL000392-formononetin (degree value = 32), respectively (Table 3, Figure 3).

The article "Combined Network Pharmacology and Molecular Docking to Verify the Treatment of Type 2 Diabetes with Pueraria Lobata Radix and Salviae Miltiorrhizae Radix" was published in 2023. Journal: Comput Math Methods Med.

### 3.5. Core Target Pathway Analysis

A total of 2015 BPs, 68 CCs, and 171 MFs of key targets were obtained by GO functional annotation, respectively (*P* < 0.05) (Figure 4). BP mainly involved response to xenobiotic stimulus, response to peptide, gland development, response to radiation, cellular response to chemical stress, response to oxygen levels, response to metal ion, response to decreased oxygen levels, response to hypoxia, and response to UV. CC is mainly membrane raft, membrane microdomain, transcription requlator complex, postsynaptic membrane, protein kinase compley, caveola, serine/threonine protein kinase complex, plasma membrane raft, cyclin-dependent protein kinase holoenzyme complex, and integral component of presynaptic membrane. MF mainly involves DNA-binding transcription factor binding, RNA polymerase I-specific DNA-binding transcription factor binding, ubiquitin-like protein ligase binding, ubiquitin protein ligase binding, phosphatase binding, kinase regulator activity, protein phosphatase binding, cyclin-dependent protein serine/threonine kinase regulator activity, G protein-coupled amine receptor activity, and G protein-coupled neurotransmitter receptor activity. The KEGG analysis results showed that a total of 136 signaling pathways were enriched (Figure 5), mainly related to response to xenobiotic stimulus, cellular response to chemical stress, response to peptide, gland development, response to oxygen levels, response to radiation, response to decreased oxygen levels, response to UV, response to metalion, response to hypoxia, response to reactive oxygen species, response to estradiol, response to oxidative stress, response to light stimulus, regulation of apoptotic signaling pathway, reproductive structure development, neuron death, reproductive system development, cellular response to oxidative stress, and cellular response to peptide. Based on the GO functional annotation and KEGG pathway enrichment analysis of these two main aspects, the RP-RS drug pair mainly treats T2DM through the synergistic effect of multiple pathways and multiple targets. Annotated map of the key target genes locations of RP-RS in T2DM-related pathways was presented in Figure 6. It was found that most of the key target genes are closely with AGE-RAGE signaling pathway in T2DM.

### 3.6. Molecular Docking Prediction of Key Targets for Active Ingredient Intervention in the Treatment of T2DM by RP-RS

The key targets predicted by network pharmacology were AKT1 (1H10), VEGFA (1BJ1), NOS3 (1M9J), PPARG (2VV4), MMP9 (1GKC), and VCAM1 (1VSC), respectively. Molecular docking results of the top 4 main active ingredients and 6 core targets are shown in Figure 7 and Table 4, respectively. The key targets were individually docked to the active compounds puerarin (Figure 8), formononetin (Figure 9), tanshinone iia (Figure 10), and luteolin (Figure 11). Using Discovery Studio 2019 software, the selected compounds were finally docked into the binding site by utilizing the LibDock modules. In addition, the docked pose with the highest LibDock Score was retained for each compound for the LibDock results. The results of molecular docking showed that MMP9 had the best binding energy (LibDock Score) to puerarin, formononetin, tanshinone iia, and luteolin (133.3540, 130.3760, 123.063, and 138.5800), VEGFA to puerarin, formononetin, tanshinone iia, and luteolin (117.1350, 90.4544, 77.7759, and 59.7402), AKT1 to puerarin, formononetin, tanshinone iia, and luteolin (79.3393, 53.2793, 61.7867, and 61.3038), NOS3 to puerarin, formononetin, and luteolin (141.9620, 115.5420, and 87.0491), VCAM1 to puerarin, formononetin, tanshinone iia, and luteolin (121.3260, 93.8531, 96.6147, and 100.627), and PPARG to formononetin and tanshinone iia (60.7435 and 87.5627), respectively, and the key targets were molecularly docked to the active compounds.

The article "Combined Network Pharmacology and Molecular Docking to Verify the Treatment of Type 2 Diabetes with Pueraria Lobata Radix and Salviae Miltiorrhizae Radix" was published in 2023. Journal: Comput Math Methods Med.

## 4. Discussion

Current research on T2DM has focused on several pathological alterations such as obesity-related insulin resistance and defective insulin secretion as well as decreased B-cell mass through B-cell apoptosis, and has a close association with inflammatory alterations, immune gene defects, and impaired mitochondrial function [20, 21]. In this way, the results of the network pharmacological analysis, i.e., the results of the potential mechanism of RP-RS for the treatment of T2DM and the results of the molecular docking of potential pharmacodynamic substances and key targets will be discussed.

In this study, a holistic analysis was performed using network pharmacology from multigene, multipassage, and multitarget, and 92 active ingredients of RP-RS for the treatment of T2DM were identified; the most important of which were puerarin, formononetin, tanshinone iia, and luteolin. The phytochemicals are estrogenically active polyphenolic nonsteroidal phytochemicals, which are commonly found in various plants. It has been shown that formononetin has therapeutic effects on diabetes, such as formononetin exhibited hypoglycemic effects in mice with tetraoxacillin-induced type 1 diabetes by inhibiting pancreatic *β*-cell apoptosis [22]. It was shown that formononetin significantly increased insulin sensitivity index, decreased HOMA-IR, and improved insulin resistance [23]. Puerarin, as its main active ingredient in the treatment of T2DM may participate in the whole process of inflammatory factor expression in type 2 diabetes patients, reduce the inflammatory response, regulate the body's internal environment, and improve the state of insulin resistance and disorders of glucose and lipid metabolism, while the symptoms of type 2 diabetes can be improved [24]. It was reported that puerarin may also ameliorated streptozotocin (STZ) pancreatic injury in mice, upregulated insulin receptor substrate 1 and insulin-like growth factor protein expression in the pancreas, inhibited STZ-induced apoptosis of islet *β*-cells in diabetic mice, and increased serum insulin levels; and its protective effects on *β*-cells may be mediated by modulating the phosphatidylinositol 3-kinase/protein kinase B pathway, thereby exerting hypoglycemic effects and improving glucose tolerance [25]. In previous study, puerarin may also upregulated the gene expression of retinal vascular endothelial growth factor and hypoxia-inducible factor-1, which had a significant protective effect against STZ-induced diabetic retinopathy in rats, while VEGF, an angiogenic and vascular permeability factor, was significantly increased in the vitreous and aqueous fluids of eyes with proliferative diabetic retinopathy [26]. In addition, tanshinone iia has been reported to antagonize endothelial damage and antioxidant effects to effectively reduce diabetic nephropathy [27] and diabetic neuropathy [28]. Previous studies have shown that luteolin inhibits high-glucose-induced activation of NF-*κ*B in human monocytes and the release of the proinflammatory factor TNF-*α*, with potential preventive and therapeutic activity in diabetes mellitus [29]. It was revealed that have a regulatory effect on endothelial cell function, and luteolin enhance insulin action in adipocytes by activating the PPAR pathway [30]. Recent studies have revealed the potential protective effect of luteolin on diabetes-related hypertension, which may significantly reduce diabetes-induced vascular complications and hypertension [31]. Therefore, these components of RP-RS may play an important role in the prevention and treatment of T2DM.

The article "Combined Network Pharmacology and Molecular Docking to Verify the Treatment of Type 2 Diabetes with Pueraria Lobata Radix and Salviae Miltiorrhizae Radix" was published in 2023. Journal: Comput Math Methods Med.

Core targets including AKT1, VEGFA, NOS3, PPARG, MMP9, and VCAM1 have been identified as important by network pharmacological analysis. AKT1 is involved in several regulatory processes, including glucose metabolism, and AKT mediates insulin signaling and interacts with the transcription factors PGC-1*α* and FoxO1 to stimulate gluconeogenic gene expression [32]. AKT is part of the insulin-signaling pathway that directly inhibits the expression of PGC-1*α* protein in hepatocytes [33]. This pathway is able to regulate lipid secretion in type 2 diabetes. Because of AKT-induced inhibition of PGC-1*α* leads to inhibition of fatty acid oxidation in the liver, promoting PGC-1*α* activity in insulin-resistant hepatocytes may be able to eliminate lipid imbalance in T2DM patients [34]. It was reported that VEGFA promotes angiogenesis, and abnormal levels of VEGFA expression can exacerbate pathological angiogenesis and the development of diabetic retinopathy [35]. It was shown that reduced local production of VEGFA in the glomeruli of diabetic mouse models promotes endothelial injury and accelerates the progression of glomerular injury. It suggests that upregulation of VEGFA in diabetic kidneys protects microvasculature from injury, while decreased VEGFA in diabetes may be detrimental [36]. The NOS3 gene is an important 21-22 kb long gene located in vascular endothelial cells and contains 26 exons and 25 introns [37]. It has been reported that endothelial cells produce more oxygen radicals and release large amounts of Ca^2+^ in the early stages of diabetes, which leads to increased intracellular flow and activation of NOS, causing more endothelial cells to be produced. The end effector molecule of B-cell damage is NO, and NO can cause apoptosis by inducing endoplasmic reticulum stress-related apoptotic factors, indirectly damaging islet cells, and affecting insulin synthesis, and the activity of NOS will be reduced in diabetic patients in the later stages, while plasma NO levels will be reduced [38]. PPARG, a member of the nuclear hormone receptor superfamily, which has an important role in controlling lipid and glucose metabolism as well as in T2DM development [39]. Previous studies have shown that high expression of PPARG levels in adipose tissue reduces plasma lipid levels, has a beneficial role in long-term glucolipid homeostasis, reduces the incidence of visceral adipose IR, and is involved in regulating the pathological process of T2DM in obese populations [40]. DM is not only a metabolic disorder, activation of innate immunity and inflammatory response play an important role in the development of diabetes and its onset. MMP9 is a vital effector molecule of inflammatory cells; it will act as a switch in acute and chronic inflammation and is presumptively concerned within the initial part of inflammation and later tissue remodeling [41]. Hyperglycemia promotes the production of proinflammatory cytokines TNF-*α* and IL-6 production, and the expression of these proinflammatory cytokines induces an increase in MMP9 expression in an autocrine and paracrine manner [42]. Studies have demonstrated that the level of MMP9 directly affects the development of diabetic nephropathy, a complication of diabetes, and that high glucose downregulates the expression of MMP9 protein, thereby affecting its proportional imbalance and also exacerbating the development of diabetic nephropathy [43]. VCAM1 is a cell adhesion molecule that is a member of the immunoglobulin superfamily, and Guillén-Gómez et al. found that urinary VCAM1 levels were significantly higher in DN patients compared to diabetic patients, which could be a marker of renal pathology in diabetic patients [44]. In addition, VCAM1 protein level was significantly correlated with T2DM complications. The enhanced induction of VCAM1 expression in endothelial cells by circulating factors may play a role in the development of atherosclerosis in diabetes [45].

The article "Combined Network Pharmacology and Molecular Docking to Verify the Treatment of Type 2 Diabetes with Pueraria Lobata Radix and Salviae Miltiorrhizae Radix" was published in 2023. Journal: Comput Math Methods Med.

Through GO functional annotation analysis of the intersection target genes, it was found that RP-RS may regulate T2DM through various BP, cellular composition CC and MF. The GO enrichment analysis showed that RP-RS exhibits efficacy mainly via xenobiotic stimulus, response to peptide, response to oxygen levels, membrane raft, membrane microdomain, transcription requlator complex, DNA-binding transcription factor binding, RNA polymerase I-specific DNA-binding transcription factor binding, ubiquitin-like protein ligase binding, etc. The KEGG pathway enrichment results revealed that a total of 136 signaling pathways were enriched, mainly related to response to xenobiotic stimulus, cellular response to chemical stress, response to peptide, gland development, response to oxygen levels, and so on. The results of molecular docking validation showed that the key components screened by network pharmacology showed stable binding to the core targets NOS3 and MMP9, among which, the docking scores of puerarin and NOS3 were the highest, followed by those of luteolin and MMP9, and the stronger the interaction, the more stable the conformation of the compounds, indicating that puerarin showed good effects in activating NOS3 and luteolin exhibited good effects in activating MMP9 pathways, respectively.

## 5. Conclusion

In conclusion, a total of 92 active ingredients of RP-RS were obtained. The active components of RP-RS mainly including puerarin, formononetin, tanshinone iia, and luteolin which are closely associated with T2DM. A total of 29 intersecting target genes was acquired between drugs (RP-RS) and diseases (T2DM). Among them, the core target genes in treatment of T2DM mainly including VEGFA, MMP9, AKT1, NOS3, VCAM1, and PPARG, respectively. In addition, puerarin showed significant anti-T2DM effects in activating NOS3 and luteolin exhibited significant anti-T2DM effects in activating MMP9 pathways, respectively. The biological function exhibits efficacy mainly via positive regulation of xenobiotic stimulus, response to peptide, response to oxygen levels, membrane raft, and membrane microdomain. The signaling pathways that exerting their therapeutic effect on T2DM mainly including response to xenobiotic stimulus, cellular response to chemical stress, response to peptide, gland development, and response to oxygen levels. From the perspective of modern molecular biology, it was confirmed that RP-RS has good therapeutic effect on T2DM, the multitarget and multipath effects of TCM may rely on its therapeutic characteristics.

The article "Combined Network Pharmacology and Molecular Docking to Verify the Treatment of Type 2 Diabetes with Pueraria Lobata Radix and Salviae Miltiorrhizae Radix" was published in 2023. Journal: Comput Math Methods Med.

## Figures and Tables

**Figure 1:** Venn diagram of intersection genes of active ingredient related targets of RP and RS with anti-T2DM targets.

**Figure 2:** Active ingredients of RP and RS with anti-T2DM target network.

**Figure 3:** Protein interaction network of RP and RS with anti-T2DM.

**Figure 4:** RP and RS prevention and treatment of T2DM gene GO enrichment analysis diagram.

**Figure 5:** KEGG pathway enrichment bar chart of the active ingredients of RP and RS preventing and treating T2DM.

**Figure 6:** Annotated map of the target genes related the main active components of RP-RS on T2DM-related signal pathways.

**Figure 7:** Heatmap of main active ingredients of RP and RS with core target genes.

**Figure 8:** Molecular docking of puerarin with core target genes. (a) VEGFA, (b) MMP9, (c) AKT1, (d) NOS3, (e) VCAM1, and respectively.

**Figure 9:** Molecular docking of formononetin with core target genes. (a) VEGFA, (b) MMP9, (c) AKT1, (d) NOS3, (e) VCAM1, and (f) PPARG, respectively.

**Figure 10:** Molecular docking of tanshinone iia with core target genes. (a) VEGFA, (b) MMP9, (c) AKT1, (d) VCAM1, and (e) PPARG, respectively.

**Figure 11:** Molecular docking of luteolin with core target genes. (a) VEGFA, (b) MMP9, (c) AKT1, (d) NOS3, and (e) VCAM1, respectively.

**Table 1:** A total of possible active ingredient information of RP and RS. (a) Intersection genes between T2DM and RS. (b) Intersection genes between T2DM and RP. (c) Intersection genes among T2DM, RP, and RS.

MOL_ID	Classification	Molecule_name	Ob	Mw	Dl
MOL000358	RP	Beta-sitosterol	36.9139058327	414.790	0.75123
MOL012297	RP	Puerarin	24.0308979964	416.410	0.69099
MOL002959	RP	3′-Methoxydaidzein	48.5690937439	284.280	0.24261
MOL004631	RP	7,8,4′-Trihydroxyisoflavone	20.6680736276	270.250	0.21583
MOL000392	RP	Formononetin	69.6738806088	268.280	0.21202
MOL000390	RP	Daidzein	19.4410626585	254.250	0.18694
MOL007140	RS	(Z)-3-[2-[(E)-2-(3,4-dihydroxyphenyl)vinyl]-3,4-dihydroxy-phenyl]acrylic acid	88.5360210103	314.310	0.25869
MOL007150	RS	(6S)-6-hydroxy-1-methyl-6-methylol-8,9-dihydro-7H-naphtho[8,7-g]benzofuran-10,11-quinone	75.3858784662	312.340	0.4551
MOL007058	RS	Formyltanshinone	73.4446220045	290.280	0.41736
MOL007120	RS	Miltionone II	71.0297032063	312.390	0.43711
MOL007105	RS	Epidanshenspiroketallactone	68.2731592943	284.380	0.30549
MOL007155	RS	(6S)-6-(hydroxymethyl)-1,6-dimethyl-8,9-dihydro-7H-naphtho[8,7-g]benzofuran-10,11-dione	65.25893771	310.370	0.44871
MOL007130	RS	Prolithospermic acid	64.3709620672	314.310	0.31017
MOL007050	RS	2-(4-hydroxy-3-methoxyphenyl)-5-(3-hydroxypropyl)-7-methoxy-3-benzofurancarboxaldehyde	62.7841472598	356.400	0.39628
MOL007068	RS	Przewaquinone B	62.2400596208	292.300	0.41374
MOL000569	RS	Digallate	61.8486180263	322.240	0.25635
MOL007081	RS	Danshenol B	57.950875299	354.480	0.55764
MOL007082	RS	Danshenol A	56.9652489923	336.410	0.52172
MOL007069	RS	Przewaquinone c	55.7416730964	296.340	0.40408
MOL007108	RS	Isocryptotanshi-none	54.9819324596	296.390	0.39449
MOL007125	RS	Neocryptotanshinone	52.4879970089	314.410	0.32306
MOL007079	RS	Tanshinaldehyde	52.4747043036	308.350	0.45196
MOL007088	RS	Cryptotanshinone	52.3419622629	296.390	0.39555
MOL007094	RS	Danshenspiroketallactone	50.4312810266	282.360	0.3067
MOL007111	RS	Isotanshinone II	49.9160257407	294.370	0.39674
MOL007154	RS	Tanshinone iia	49.8873000352	294.370	0.39781
MOL007119	RS	Miltionone I	49.6843943314	312.390	0.32125
MOL007098	RS	Deoxyneocryptotanshinone	49.4003470541	298.410	0.28555
MOL007048	RS	(E)-3-[2-(3,4-dihydroxyphenyl)-7-hydroxy-benzofuran-4-yl]acrylic acid	48.2436324414	312.290	0.31229
MOL007156	RS	Tanshinone VI	45.6373060194	296.340	0.29549
MOL007141	RS	Salvianolic acid g	45.5648557799	340.300	0.60602
MOL001942	RS	Isoimperatorin	45.4642467387	270.300	0.22524
MOL007115	RS	Manool	45.0443163606	304.570	0.20208
MOL007101	RS	Dihydrotanshinone I	45.0432791888	278.320	0.36015
MOL007123	RS	Miltirone II	44.9510664818	272.320	0.23537
MOL007045	RS	3*α*-hydroxytanshinone II A	44.92933597	310.370	0.44272
MOL001659	RS	Poriferasterol	43.8298515785	412.770	0.75596
MOL002651	RS	Dehydrotanshinone II A	43.7622859945	292.350	0.40019
MOL007077	RS	Sclareol	43.6706845842	308.560	0.2058
MOL007152	RS	Przewaquinone E	42.8548520397	312.340	0.45301
MOL007151	RS	Tanshindiol B	42.6658104891	312.340	0.45303
MOL007070	RS	(6S,7R)-6,7-dihydroxy-1,6-dimethyl-8,9-dihydro-7H-naphtho[8,7-g]benzofuran-10,11-dione	41.3104570553	312.340	0.453
MOL007041	RS	2-isopropyl-8-methylphenanthrene-3,4-dione	40.8601540814	264.340	0.22897
MOL007071	RS	Przewaquinone F	40.3078839947	312.340	0.45925
MOL002776	RS	Baicalin	40.1236099599	446.390	0.75264
MOL007118	RS	Microstegiol	39.6122945749	298.460	0.27734
MOL006824	RS	*α*-Amyrin	39.5120897831	426.800	0.76221
MOL007124	RS	Neocryptotanshinone II	39.4629911416	270.350	0.23157
MOL007093	RS	Dan-shexinkum D	38.8830210096	336.410	0.55453
MOL007122	RS	Miltirone	38.7569863502	282.410	0.25418
MOL001601	RS	1,2,5,6-Tetrahydrotanshinone	38.7453867227	280.340	0.35791
MOL007100	RS	Dihydrotanshinlactone	38.6847682981	266.310	0.32227
MOL007063	RS	Przewalskin A	37.1065006596	398.490	0.64901
MOL007061	RS	Methylenetanshinquinone	37.07319368	278.320	0.36017
MOL001771	RS	Poriferast-5-en-3beta-ol	36.9139058327	414.790	0.75034
MOL007121	RS	Miltipolone	36.5561120639	300.430	0.36803
MOL000006	RS	Luteolin	36.1626293429	286.250	0.24552
MOL002222	RS	Sugiol	36.113534855	300.480	0.27648
MOL007107	RS	C09092	36.069489858	286.500	0.2474
MOL007127	RS	1-methyl-8,9-dihydro-7H-naphtho[5,6-g]benzofuran-6,10,11-trione	34.7208221315	280.290	0.36634
MOL007149	RS	NSC 122421	34.4929230859	300.480	0.27645
MOL007049	RS	4-Methylenemiltirone	34.348675885	266.360	0.22726
MOL007036	RS	5,6-dihydroxy-7-isopropyl-1,1-dimethyl-2,3-dihydrophenanthren-4-one	33.7652523626	298.410	0.28585
MOL007143	RS	Salvilenone I	32.4347085631	270.400	0.22895
MOL007059	RS	3-beta-Hydroxymethyllenetanshiquinone	32.1610337648	294.320	0.40894
MOL007145	RS	Salviolone	31.7241503895	268.380	0.23568
MOL007085	RS	Salvilenone	30.3836538737	292.400	0.37639

The article "Combined Network Pharmacology and Molecular Docking to Verify the Treatment of Type 2 Diabetes with Pueraria Lobata Radix and Salviae Miltiorrhizae Radix" was published in 2023. Journal: Comput Math Methods Med.

**Table 2:** Main ingredients from RP and RS based on number of corresponding targets. (a) PPI visualization network diagram of 120 targets; (b) PPI visualization network diagram of 29 core targets.

MOL_ID	Molecule_name	Classification	Ob	Mw	Dl
MOL012297	Puerarin	RP	24.0308979964	416.410	0.69099
MOL000392	Formononetin	RP	69.6738806088	268.280	0.21202
MOL007154	Tanshinone iia	RS	49.8873000352	294.370	0.39781
MOL000006	Luteolin	RS	36.1626293429	286.250	0.24552

**Table 3:** Corresponding core targets genes of main ingredient based on the degree value.

Gene name	Degree	Betweenness centrality	Closeness centrality
AKT1	26	0.09722044	0.93333333
VEGFA	25	0.08297252	0.90322581
NOS3	24	0.0748313	0.875
PPARG	22	0.06089927	0.82352941
MMP9	22	0.04616644	0.82352941
VCAM1	20	0.04275445	0.77777778
CAT	20	0.0317474	0.77777778
STAT3	19	0.0224157	0.75675676
IL4	18	0.02462019	0.73684211
HIF1A	16	0.00700457	0.7
CTNNB1	16	0.01164871	0.7
ESR1	15	0.01381435	0.68292683
TGFB1	15	0.0043485	0.68292683
SIRT1	14	0.00583073	0.66666667
GPT	13	0.00790826	0.65116279
NOS2	13	0.00240188	0.65116279
SOD1	10	0.00254587	0.60869565
AGTR1	10	0.00472411	0.60869565
DPP4	10	0.00459492	0.60869565
AR	9	0.00176367	0.58333333
SELP	9	0.00262661	0.59574468
CD40LG	7	0	0.57142857
AKR1B1	7	7.94E-04	0.57142857
ACE2	7	6.42E-04	0.57142857
CYP19A1	6	5.93E-04	0.56
LEPR	6	1.89E-04	0.56
PLAT	5	0	0.54901961
PON1	5	2.04E-04	0.53846154
ADRB2	5	2.94E-04	0.54901961

The article "Combined Network Pharmacology and Molecular Docking to Verify the Treatment of Type 2 Diabetes with Pueraria Lobata Radix and Salviae Miltiorrhizae Radix" was published in 2023. Journal: Comput Math Methods Med.

**Table 4:** The results of molecular docking.

Compound	Target	PDB	LibDock score
Puerarin	VEGFA	1BJ1	117.1350
Puerarin	MMP9	1GKC	133.3540
Puerarin	AKT1	1H10	79.3393
Puerarin	NOS3	1M9J	141.9620
Puerarin	VCAM1	1VSC	121.3260
Puerarin	PPARG	2VV4	0
Formononetin	VEGFA	1BJ1	90.4544
Formononetin	MMP9	1GKC	130.3760
Formononetin	AKT1	1H10	53.2793
Formononetin	NOS3	1M9J	115.5420
Formononetin	VCAM1	1VSC	93.8531
Formononetin	PPARG	2VV4	60.7435
Tanshinone iia	VEGFA	1BJ1	77.7759
Tanshinone iia	MMP9	1GKC	123.0630
Tanshinone iia	AKT1	1H10	61.7867
Tanshinone iia	NOS3	1M9J	0
Tanshinone iia	VCAM1	1VSC	96.6147
Tanshinone iia	PPARG	2VV4	87.5627
Luteolin	VEGFA	1BJ1	59.7402
Luteolin	MMP9	1GKC	138.5800
Luteolin	AKT1	1H10	61.3038
Luteolin	NOS3	1M9J	87.0491
Luteolin	VCAM1	1VSC	100.627
Luteolin	PPARG	2VV4	0

## Data Availability

The data that support the findings of this study are available from the corresponding authors upon reasonable request.

## Abbreviations

RP: *Pueraria Lobata Radix*
RS: *Salviae Miltiorrhizae Radix*
RP-RS: *Pueraria Lobata Radix* (RP) and *Salviae Miltiorrhizae Radix*
T2DM: Type 2 diabetes mellitus
TCMSP: Traditional Chinese medicine system pharmacology
GO: Gene Ontology
KEGG: Kyoto Encyclopedia of Genes and Genomes
PPI: Protein-protein interaction
TCM: Traditional Chinese medicine
DM: Diabetes mellitus
OB: Bioavailability
DL: Drug-like properties
BP: Biological process
CC: Cellular component
MF: Molecular function
STZ: Streptozotocin.
